# *Aedes albopictus* salivary proteins adenosine deaminase and 34k2 interact with human mast cell specific proteases tryptase and chymase

**DOI:** 10.1080/21655979.2022.2081652

**Published:** 2022-06-23

**Authors:** Zhiqiang Li, Cejuan Ji, Jinzhi Cheng, Magnus Åbrink, Tao Shen, Xiaoyuan Kuang, Zhengling Shang, Jiahong Wu

**Affiliations:** a The Key and Characteristic Laboratory of Modern Pathogen Biology, College of Basic Medicine, Guizhou Medical University, Department of Medical Parasitology, College of Basic Medicine, Guizhou Medical University, Guiyang, Guizhou, China; b Department of Medical Technology, Guiyang Healthcare Vocational University, Guiyang, Guizhou, China; c Department of Immunology, College of Basic Medicine, Guizhou Medical University, Guiyang, Guizhou, China; d Section of Immunology, Department of Biomedical Sciences and Veterinary Public Health, Swedish University of Agricultural Sciences, Uppsala, Sweden

**Keywords:** *Aedes albopictus*, adenosine deaminase, 34k2, mast cell, tryptase, chymase

## Abstract

When mosquitoes probe to feed blood, they inoculate a mixture of salivary molecules into vertebrate hosts’ skin causing acute inflammatory reactions where mast cell-derived mediators are involved. Mosquito saliva contains many proteins with largely unknown biological functions. Here, two *Aedes albopictus* salivary proteins – adenosine deaminase (alADA) and al34k2 – were investigated for their immunological impact on mast cells and two mast cell-specific proteases, the tryptase and the chymase. Mouse bone marrow-derived mast cells were challenged with increased concentrations of recombinant alADA or al34k2 for 1, 3, and 6 h, and to measure mast cell activation, the activity levels of β-hexosaminidase and tryptase and secretion of IL-6 were evaluated. In addition, a direct interaction between alADA or al34k2 with tryptase or chymase was investigated. Results show that bone marrow-derived mast cells challenged with 10 μg/ml of alADA secreted significant levels of β-hexosaminidase, tryptase, and IL-6. Furthermore, both al34k2 and alADA are cut by human tryptase and chymase. Interestingly, al34k2 dose-dependently enhance enzymatic activity of both tryptase and chymase. In contrast, while alADA enhances the enzymatic activity of tryptase, chymase activity was inhibited. Our finding suggests that alADA and al34k2 via interaction with mast cell-specific proteases tryptase and chymase modulate mast cell-driven immune response in the local skin microenvironment. alADA- and al34k2-mediated modulation of tryptase and chymase may also recruit more inflammatory cells and induce vascular leakage, which may contribute to the inflammatory responses at the mosquito bite site.

## Highlights

- Aedes albopictus saliva causes mast cell degranulation.
- ADA, but not 34k2, induces mast cell degranulation and secretion of tryptase and IL-6.
- ADA and 34k2 are cleaved by recombinant human tryptase and chymase
- Both ADA and 34k2 modulates the enzymatic activities of recombinant human tryptase and chymase

## Introduction

*Aedes albopictus*, also known as the Asian tiger mosquito, belongs to the order Aedes genera, family Culicidae, Diptera. This highly invasive species can be found in many parts of the world and as it can resist long-term desiccation and abide in colder weather *Ae. albopictus* is predicted to a dramatic global expansion [1]. Furthermore, the aggressive ‘bite’ behavior and induced inflammatory responses by *Ae. albopictus* mosquitoes not only decrease the happiness of the public but also may contribute to the transmission of several arboviruses such as Zika virus, West Nile virus, and dengue virus [2–4].

During the probing and before blood feeding, female *Ae. albopictus* mosquitoes insert their mouthparts into the host skin and then make several attempts to locate the blood vessel [5]. In the probing process, a cocktail of salivary proteins secreted from mosquito salivary gland is injected into the skin. This injection will ignite immune responses causing immediate cutaneous reactions and delayed inflammatory responses with symptoms of itching, swelling, redness, and pain at the mosquito bite site [6,7]. An early study demonstrated that mosquitoes with their salivary glands removed still were able to do probing but no skin reactions were observed [8], suggesting an essential role of injected saliva for the development of cutaneous reactions. Salivary components were found to exert pharmacological functions by acting as anti-inflammatory, antiplatelet, anticoagulant molecules, and vasodilators [7]. Salivary proteins of *Ae. albopictus* mosquitoes with high immunogenicity triggered production of IgE and IgG antibodies [9] and the D7 long form protein could inhibit platelet aggregation and recruitment of neutrophils and eosinophils [7]. Furthermore, *Ae. albopictus* has via two novel allergens *Aed al 2* and *Aed al 3* been reported to induce allergic responses associated with IgE [10,11]. However, relatively few studies to identify and characterize the biological functions of *Ae. albopictus* salivary proteins have been executed.

Mast cells play important roles during immune responses especially in innate immunity. There are two human mast cell subclasses, the ‘MC_T_’ type expressing tryptase only, and the ‘MC_TC_’ type expressing tryptase, chymase, and carboxypeptidase A3. The MC_TC_ resides close to blood vessels, nerves, smooth muscles and hair follicles in skin. Upon activation leading to degranulation mast cells release large quantities of preformed mediators, including the mast cell-specific proteases tryptase and chymase [12,13]. These two proteases have been reported to be involved in many diseases, e.g. allergy-associated reactions [14]. The tryptase level in serum can be used as a biomarker for mast cell-associated disorders [12], and tryptase shows a significant role in epithelial wound healing [15], whereas chymase, for example, has a major impact on the phenotype of human lung fibroblasts and the bronchial epithelium integrity [16,17].

In mosquito bite-induced cutaneous reactions, mast cells were reported to play essential roles, and they increased at the *Aedes aegypti* mosquito bite sites [18]. In studies with *Anopheles gambiae* and *Anopheles stephensi* bitten mice, mast cell degranulation was observed [6,19]. Furthermore, mast cell degranulation could be directly triggered by *Anopheles stephensi* saliva, whereas mast cell deficiency decreased the inflammatory infiltrate and vascular permeability at bitten skin sites [19], and *Ae. albopictus* bite-induced itching was caused by histamine released from mast cells [20]. Although many mosquito allergens identified in mosquito bite or saliva gland extracts generate IgE and IgG antibody responses in the host, very few studies have been done to characterize the impact of mosquito saliva proteins on mast cells or the mast cell-specific proteases tryptase and chymase.

Here, we investigated the potential roles of two proteins from *Ae. albopictus* saliva: adenosine deaminase (alADA) and al34k2. We cloned, expressed and purified these two proteins, and then used them to challenge mouse bone marrow-derived mast cells and in interaction studies with recombinant human chymase and human skin tryptase. We demonstrate that alADA caused mast cell degranulation, and that both alADA and al34k2 modulated tryptase and chymase enzymatic activities. Furthermore, both alADA and al34k2 were degraded by the two mast cell proteases. Our study highlights the potential roles of alADA and al34k2 in mast cell-driven inflammatory responses after *Ae. albopictus* mosquito bite. Future perspectives will focus on investigating the potential roles of alADA and al34k2 in inflammation and pathogen transmission *in vivo*, using mast cell protease-4 (*Mcpt*4, similar to human chymase) or mast cell protease-6 (*Mcpt*6, similar to human tryptase) gene knockout mice.

The aim of this study was to investigate the impact of alADA and al34k2 on mast cells and the mast cell-specific proteases tryptase and chymase, and the goal was to demonstrate that alADA and al34k2 could exert immunomodulatory roles via functional interactions with the mast cell proteases.

## Materials and methods

### Animals

Balb/c mice were kept under the permission NO. 2,000,050 granted from Guizhou Medical University Experimental Animal Center. Bone marrow for generation of bone marrow mast cells was obtained from the tibia and femur bone of 8–10 weeks old in house-bred Taconic mice. All mice were treated with high humanity and housed in enriched environment in Department of Immunology, College of Basic Medicine, Guizhou Medical University.

### *Preparations* of Ae. Albopictus *saliva and soluble thoraxes proteins*

*Ae. albopictus* mosquitoes were fed with fresh 10% sugar dissolved in sterile water and reared at 26 ± 1°C and a light:dark (14:10) photoperiod in the mosquito room of The Key and Characteristic Laboratory of Modern Pathogen Biology, College of Basic Medicine, Guizhou Medical University. To get mosquito saliva, more than 200 adult female mosquitoes were fed with 500 μl of fresh 10% sugar filled in a cap of 50-ml Falcon tube, 24 h later, sugar containing mosquito saliva was collected. This process was repeated until getting 2 ml of saliva. The protein concentration was determined with BCA protein assay kit (Meilunbio, #MA0082, China), where after the collected saliva was sterile filtered through a 0.22-μm filter. The sterile *Ae. albopictus* saliva was stored at −80°C until used.

To get soluble salivary gland proteins, 10 *Ae. albopictus* female mosquitoes in a cell culture dish were placed for 1 min in −20°C, where after thoraxes were dissected out with two fine-tipped tweezers. The pooled thoraxes resuspended in 500 μl phosphate-buffered saline were disrupted using a tissue homogenizer, and the homogenate centrifuged at 8000 rpm for 5 min. The supernatant was kept in −80°C until used.

### Staining of SDS-PAGE gels with Coomassie blue

Salivary protein samples were analyzed on SDS-PAGE gels according to standard procedures. Gels were stained in Coomassie blue buffer (0.1% Coomassie brilliant blue R-250, 50% methanol and 10% Acetic acid) overnight, and then de-stained in buffer (10% acetic acid, 40% EtOH, and 50% sterile H_2_O) for 40 min with three to four changes. Photos of the de-stained gels were taken with the ImageQuant 400 imaging system.

### Protein identification

The protocol was performed as described in Ref. [21]. The proteins bands marked with numbers 1, 2, and 3 in Supplementary Figure 1 were individually excised from gel, cut into 1–2 mm^3^ pieces and detained in 50% acetonitrile (ACN) containing 100 mM NH_4_HCO_3_ (pH 8.0) at room temperature. The gel pieces were washed twice in 100% ACN and then dried in a micro-centrifugal vacuum concentrator. Then, 10 mM of dithiothreitol in 50 mM NH_4_HCO_3_ (pH 8.0) was added and incubated with the gel pieces at 56°C for 60 min. After washing in ACN twice, the gel pieces were then incubated with 60 mM iodoacetic acid in 50 mM NH_4_HCO_3_ (pH 8.0) in the dark for 45 min. Excessive solution was discarded, and then wash step was repeated twice in ACN. Gel pieces were dried and then treated with 15 ng/µL of trypsin in NH_4_HCO_3_ followed by incubation at 37°C overnight. The supernatant of the tryptic digest was collected, and the remaining peptides were extracted three times in ACN containing 0.1% formic acid.

The mass spectrometry was performed using the Q Exactive™ Hybrid Quadrupole-Orbitrap Mass Spectrometer from Thermo Scientific (LC-MS/MS). Peptides were injected into autosampler and trapped in C18 column (3 µm particle size, 75 μm × 20 mm,100 Å pore size). The peptides were then eluted on a reversed phase capillary column (2 μm particle size, 50 μm × 150 mm, 100 Å pore size, Thermo). Two mobile phases (solvent A: 99% H_2_O, 0.1% formic acid and solvent B: 80% ACN, 0.1% formic acid) were set to establish a 100-min analytical gradient (0 min in 3% B, 0–5 min of 3–5% B; 5–70 min of 5–23% B, 70–90 min of 23–60% B, 90–92 min of 60–90% B, 90% B for 8 min). The flow rate of the liquid phase was set at 300 nL/min. Each scan cycle contained a MS full scan (*m*/*z* range was 350–1800, ion accumulation was 200 ms), followed by 40 MS/MS scans (*m*/*z* range was 100–1500, ion accumulation was 50 ms). MS/MS acquisition conditions were set that the parent ion signal was more than 3e6 and the charge number was +2 to +5.

The data generated by LC-MS/MS were searched using Protein Discover (V2.2). The database used for search was the *Aedes albopictus* database (uniprot-aedes + albopictus + organism __ Aedes+albopictus_. fasta) in UniProt proteomic reference database. The retrieval parameters were as follows: Scan Event: Msaa Analyzer (FTMS), MS Order (MS2), Activation Type (HCD), scan typr (full); Sequest HT: Enzyme (Trypsin full), Dynamic Modification (Oxdation, Acetyl, Carbamidomethyl). Maximum Delta Cn and Maximum Rank of Propensity Score Match were set ≥0.05 as the standard to screen the data. The items and contaminated proteins retrieved from the reverse database were deleted, and the remaining identification information was used for subsequent analysis.

### Cloning, expression, and purification of alADA and al34k2

The protocol was performed as described in Ref. [22]. In brief, the cDNA was synthesized with total RNA obtained from 10 female *Ae. albopictus* mosquito thoraxes using PrimerScript RT Reagent Kit (TaKaRa, #RR037B). The sequences of alADA (GenBank: AAV90660.1) and al34k2 (GenBank: AY826118.1) were used to design the specific primers. The amplification of alADA was performed with nested PCR by using the forward primer 1(F1) 5′- CGC GGA TCC GAC GAC GAC GAC AAG CAA CAT CTT ATT ACA TCA AGC-3′ (BamHI), F2 5′- CGC GAC GAC AAG AGC CCA TCC CTC CCG GAG AGC-3′, and reverse primer (R) 5′- CCG CTC GAG TCA CAC GAT TTT CAT AAT CC-3′ (XhoI). The sequence of al34k2 was amplified using F1 5′- CTA GGA TCC ATG AAG ACT TCT CTT CCG ATA GTC-3′ (BamHI), F2 5′- CTA GGA TCC AAC CCA ACC CCA AAG TCG TGC AC-3′, and R 5′- CGT CCT CGA GTT AAC CGA ATC TGA TGG TGA CC-3′ (XhoI). The amplified PCR products were cloned into pMD18-T vector and then subcloned into pET28a (+) vector (TaRaKa). The resulting recombinant alADA or al34k2 plasmids were transformed into *Escherichia coli* BL21 (DE3) at 37°C and then the 1 mM isopropyl-β-D-thiogalactosidase was added to incubate for 5 h. Finally, recombinant alADA and al34k2 were purified with His•Bind Purification Kit (Novagen). The absence of endotoxin was tested using ELISA Kit for Lipopolysaccharides (#SEB526Ge, Cloud-Clone Corp, China).

### Western blotting

Western blotting was performed as described [23]. Briefly, 15 μg of purified alADA or al34k2 was transferred from 12% SDS-Page gel to PVDF membranes. The membranes were blocked with blocking buffer (5% skim milk in Tris-buffer saline Tween-20) overnight, and incubated with mouse anti-alADA and anti-al34k2 serum diluted 1:100, respectively, at 4°C overnight. After incubation with the primary sera membranes were washed twice in washing buffer (Tris-buffer saline) and incubated with a 1:2000 diluted secondary horseradish peroxidase-conjugated goat anti-mouse IgG antibody (Sigma-Aldrich), at 37°C for 60 min. The immunoblots were examined by an Enhanced Chemiluminescence Substrate Kit (Thermo Fisher Scientific, Waltham, MA, USA).

### Bone marrow derived mast cells: preparation, culture, and in vitro stimulation

To obtain bone marrow-derived mast cells (BMMCs), bone marrow was isolated from femur and tibia of mice as described in Ref. [24]. Cells were washed twice with PBS and cultured in complete Roswell Park Memorial Institute (RPMI) 1640 medium supplemented with 10% FCS, 1% PEST, 1% mercaptoethanol, 5% nonessential amino acid, 20 ng/ml of recombinant murine SCF (Peprotech, #250-03) and 20 ng/ml of IL-3 (Peprotech, #213-13). After 3 to 4 weeks, mast cells were verified with May–Grünwald/Giemsa staining. The BMMCs were washed three times with PBS and seeded in 24 well plates at 1 × 10^6^ cells per ml in serum-free HBSS and stimulated with different concentrations (10, 100, or 1000 ng/ml) of mosquito salivary proteins for 6 h. In addition, cultures of 1 × 10^6^ BMMCs per ml in serum-free HBSS were challenged with 0.1, 1.0, and 10 μg/ml of alADA for 3 and 6 h, or al34k2 for 1 h and 6 h. The supernatants were collected and kept at −80°C until used.

### Measurement of β-hexosaminidase and tryptase activities

For the measurement of β-hexosaminidase activity, we followed the protocol as previously described [24]. Briefly, 80 μl of cell supernatants were incubated with 20 μl of 5 mM *p*-nitrophenyl *N*-acetyl β-D-glucosamine (Absin, #abs42136928) dissolved in citrate buffer for 1 h at room temperature. After adding of 200 μl 0.05 M sodium carbonate reaction buffer, the optical density was measured at 405 nm.

For the tryptase assay, 80 μl of cell supernatants were incubated with 20 μl of the 2.5 mM substrate S-2288 (H-D-Ile-Pro-Arg-pNA, Chromogenic, Sweden), for overnight at ambient temperature. The absorbance at 405 nm was determined at time points 0 and 24 h, and the difference in optical density was calculated.

### IL-6 detection by ELISA assay

IL-6 level in cell supernatants was determined using Mouse IL-6 DuoSet ELISA Kit (R&D, #DY406-05), according to manufacturer’s protocol.

### Degradation assay of alADA and al34k2

To analyze mast cell protease-mediated degradation of alADA and al34k2, 20 μg alADA or al34k2 was mixed with 0.2–2 μg of recombinant human tryptase (rHT, #G706A, Promega) or with 0.002 to 0.02 μg chymase (rHC, #C8118-50UG, Sigma). At room temperature, the degradation was allowed to proceed for 1 h to overnight for rHT, and for 10, 30, or 60 min for rHC. alADA or al34k2 alone was incubated as a control. Electrophoresis and Coomassie blue staining were performed to visualize the enzymatic degradation of the alADA or al34k2. A chymase inhibitor HY-109059 (Fulacimstat, # HY-109059, MedChemExpress) was used to show chymase-specific degradation of alADA and al34k2.

### Detection of the effect of alADA and al34k2 on mast cell proteases activity

In tryptase and chymase activity assays the salt concentration of the buffer can affect the result [24]. Here, we used sterile PBS (0.15 M NaCl) as the dilution and reaction buffer. To test if alADA and al34k2 had an effect on tryptase or chymase activity, different amounts of the mosquito proteins, i.e. 0.01, 0.1, 1, or 10 μg of alADA or al34k2, were incubated with 0.02 μg of rHT or 0.01 μg of rHC in a final total volume of 100 μl PBS. At room temperature 20 μl of the 2.5 mM substrates, S-2288 for tryptase and L-1595 for chymase were added, and the optical density (OD) at 0, 10, 30, 40, and 60 min was measured at 405 nm. The OD comparisons among five groups at different time points were statistically analyzed. Three independent experiments were performed, each experiment was done in triplicate.

### Statistical analysis

Statistical analysis of data was performed with GraphPad Prism 8 using the non-parametric Welch’s *t* test. *P* values ≤0.05 represents significant differences between compared groups.

## Results

In this study, we examined the interactions of *Ae. albopictus* salivary proteins, focusing mainly on alADA and al34k2, with the mast cell-specific proteases tryptase and chymase, to explore the potential roles of alADA and al34k2 in modulating the immune responsive environment at the mosquito bite sites. We demonstrated alADA and al34k2 exert immunomodulatory roles via interaction with mast cell tryptase and chymase *in vitro*.

### *Ae. albopictus* saliva cause mast cell degranulation

Mast cell degranulation was observed in *Anopheles stephensi* bitten mice [6] indicating that mast cells may also degranulate in response to *Ae. albopictus* saliva. Thus, to examine if there is a direct interaction between mast cells and *Ae. albopictus* saliva we initially challenged bone marrow-derived mast cells (BMMCs) with increased concentrations of *Ae. albopictus* saliva. As a readout of mast cell degranulation, beta-hexosaminidase activity was determined in the BMMC supernatants. Direct exposure of BMMCs with *Ae. albopictus* saliva increased the activity of beta-hexosaminidase significantly (Figure 1), suggesting that mast cells degranulate in response to the mosquito saliva.

**Figure 1.** ***Aedes Albopictus* saliva induces degranulation of mouse bone marrow-derived mast cells (BMMCs)**. To determine if *Aedes Albopictus* saliva activates mast cells 1 × 10^6^ BMMCs seeded in 1 ml HBSS were challenged with three concentrations, 10 ng/ml, 100 g/ml, and 1000 ng/ml, of the collected *Aedes Albopictus saliva*. Beta-hexosaminidase activity (a with *N* = 3) was determined in supernatants collected at 6 h. Data are pooled from two independent experiments with BMMCs derived from a total of three individual mice. In duplicate cultures. Data are shown as mean ± SD and statistical analysis conducted by Welch’s t test with significant difference presented as *, *P* < 0.05 versus un-challenged control.

### alADA, but not al34k2, induces mast cell degranulation and secretion of tryptase and IL-6

Previous studies suggested that alADA and al34k2 of *Ae. albopictus* salivary proteins have important functions [25–28]. Therefore, we cloned, expressed and purified these two proteins (Figures 2a, 2b) to investigate if they could activate mast cells. BMMCs were challenged with three concentrations (0.1, 11.0,or 10 μg/ml) of the recombinant proteins alADA or al34k2. Beta-hexosaminidase activity, tryptase activity and IL-6 levels were determined in supernatants collected at different time points, i.e. 1 and 3 h for al34k2, or 3 and 6 h for alADA. The challenge with al34k2 did not induce significantly changed beta-hexosaminidase, tryptase and IL-6 levels (Figures 3a, 3b). In contrast, BMMCs challenged with 10 μg/ml of alADA showed a significantly increased release of beta-hexosaminidase, ttryptase,and IL-6 (Figures 3c, 3d). Together, our data suggest that alADA, but not al34k2, cause mast cell activation and degranulation.

**Figure 2.** **Visualization of purified alADA and al34k2**. alADA and al34k2 were cloned and expressed. The purified was visualized on 12% SDS-PAGE gel using Coomassie blue staining.

**Figure 3.** **alADA, but not al34k2 induces degranulation and secretion of tryptase and IL-6 from mouse bone marrow-derived mast cells (BMMCs)**. To determine if alADA and al34k2 activate mast cells 1 × 10^6^ BMMCs seeded in 1 ml HBSS were challenged with three concentrations, 0.1 , 1,and 10 μg/ml, of the recombinant proteins alADA or al34k2. Beta-hexosaminidase activity, tryptase activity and IL-6 were determined in supernatant collected at time points 1 or 3 h for al34k2, 3 or 6 h for alADA. Data are pooled from three independent experiments with BMMCs derived from a total of three individual mice. In duplicate cultures. Data are shown as mean ± SE and statistical analysis conducted by Welch’s *t* test with significant difference presented as * *P* < 0.05, **P < 0.01 versus un-challenged control.

### Both alADA and al34k2 can be cleaved by recombinant human tryptase and chymase

To further investigate the potential interactions between alADA or al34k2 and the mast cell-specific proteases, *Ae. albopictus* salivary proteins were assayed for degradation by recombinant human tryptase (rHT) and chymase (rHC). Soluble salivary gland proteins purified from *Ae. albopictus* thoraxes were incubated overnight with either rHT (S Figure 1a) or rHC (S Figure 1b). Several degraded protein bands were observed and the proteomics analysis found alADA among identified proteins possibly cleaved by rHT or/and rHC (S Figure 2). The protein sequences of alADA and al34k2 were screened for the rHT and rHC extended target sites, and as shown in (Figures 4a, 4b), both alADA and al34k2 contain four rHC target sites, as well as eight and three rHT target sites, respectively. This suggested that alADA and al34k2 could be cleaved by rHT and rHC, and incubation with different concentrations of rHT or rHC for different hours showed significant degradation (Figures 5, 6). The incubation with a high concentration of rHT showed complete degradation of alADA (overnight) and a significant cleavage of alADA after 3 and 6 h (Figure 5a), whereas rHT progressively cleaved al34k2 into smaller peptides (Figure 5b). Furthermore, at 0.2 μg concentration of rHC alADA was clearly cleaved (Figure 6a, b), whereas 0.02 μg of rHC sufficiently degraded al34k2 (Figure 6c, d). The chymase inhibitor HY-109059 significantly reduced the degradation of alADA and al34k2 (Figure 6b, 6d). Collectively, our data suggest that alADA and al34k2 have a direct interaction with rHT and rHC, thus indicating that these mast cell proteases can limit the biological functions of alADA and al34k2.

**Figure 4.** **The physiologic target sites of alADA and al34k2 for rHT and rHC**. Tryptase prefers to cut after K) or R in its three amino acid target sites (K/R + X + K/R). The physiologic target sites for chymase is eight amino acids long (P4, P3, P2, P1, P1’, P2’, P3’, P4’). Chymase preferentially cuts after aromatic amino Y or F, W located in the P1 position and requires E or D in the P2’ position. alADA (a) and al34k2 (b) contain four rHT target sites, and have eight and three rHC target sites, respectively.

**Figure 5.** **Both alADA and al34k2 can be cleaved by rHT**. To determine if rHT can degrade alADA and al34k2, 20 μg of alADA (a) or al34k2 (b) was incubated with three different coccentrations of rHT for different time points.

**Figure 6.** **rHC can cleave alADA and al34k2**. To examine if alADA and al34k2 can be degraded by rHC, 20 μg of alADA or al34k2 was incubated with different concentrations of rHC for different time points (a, c) as shown in the figure. A chymase inhibitor HY-109059 was used to investigate the degradation ability of chymase to alADA (b) and al34k2 (d).

### Both alADA and al34k2 can modulate the enzymic activities of rHT and rHC

Previously, we found that excretory secretory protein proteins released from *Giardia intestinalis* could exert immunologic roles via modulation of mast cell tryptase and chymase enzymatic activities [24]. We therefore examined if alADA or al34k2 had modulatory effects on the enzymatic activities of rHT and rHC. Surprisingly, al34k2 dose-dependently enhanced the enzyme activities of both rHT and rHC (Figure 7a, 7c), with a significant effect on the conversion rate over 60 min of both the S-2288 and the L-1595 substrates (Figure 7b, 7d). Similarly, alADA also had a dose-dependent enhancement effect on the rHT activity (Figure 8a), even at the lowest concentrations of alADA (Figure 8b). In contrast, low concentrations of alADA had no effect on the substrate conversion rate, whereas the addition of 10 μg alADA inhibited the rHC activity up to 30 min (Figure 8c). The L-1595 substrate conversion rate decreased up to 10 min after addition of alADA, then switched from a decreased to an increased conversion rate (Figure 8d). This result suggests that the substrate conversion rate could be affected by rHC-mediated degradation of alADA. Note that alADA or al34k2 alone had no detectable effects on the substrates S-2288 and L-1595. Collectively, our data indicate that al34k2 and alADA can modulate the activities of rHT, possibly affecting the stability of the tryptase tetramer, and of rHC (Figure 7a, 8a).

**Figure 7.** **Al34k2 enhances the enzyme activity of rHT and rHC**. Four different concentrations (0.01, 0.1, 1, 10 μg) of al34k2 were incubated with 0.02 μg of rHT or 0.01 μg of rHC. The change in optical density (OD) was measured at 405 nm after adding the substrates, S-2288 (s) for tryptase (a), L-1595 (l) for chymase (c). The OD comparisons among five groups at time point 60 min were statistically analyzed (a, c). A representative experiment out of 3 independent experiments is shown. The enzyme activity rate (b for a, d for c) was determined as milli-delta OD per minute. Note that al34k2 alone has no detectable activity to S-2288 and L-1595. Data are shown as mean ± SD and statistical analysis conducted by Welch’s *t* test with significant difference presented as * *P* < 0.05, **P < 0.01, ***P < 0.01, ****P < 0.001 versus vehicle control.

**Figure 8.** **alADA modulates the enzyme activity of rHT and rHC**. 0.01, 0.1, 1, and 10 μg of alADA were incubated with 0.02 μg of rHT or 0.01 μg of rHC. The change in optical density (OD) was measured at 405 nm after adding the substrates, S-2288 (s) for tryptase (a), L-1595 (l) for chymase (c). The OD comparisons among five groups at time points 10, 30, and 60 min were statistically analyzed (a, c). Each sample was tested in triplicate, a representative experiment out of three independent experiments is shown. The enzyme activity rate (b for a, d for c) was determined as milli-delta OD per minute. Note that alADA alone has no detectable activity to S-2288 and L-1595. Data are shown as mean ± SD and statistical analysis conducted by Welch’s *t* test with significant difference presented as *P < 0.05, **P < 0.01, ***P < 0.01, ****P < 0.001 versus vehicle control.

## Discussion

Previous studies have indicated that mast cells play an important role in mosquito bite-induced inflammation. However, it remains unknown if *Ae. albopictus* bite induces mast cell activation *in vivo* and, the potential interactions of *Ae. albopictus* salivary proteins with mast cell tryptase and chymase have not been explored. To this end we studied the potential interactions between mosquito saliva and mast cells using mouse bone marrow-derived mast cells (BMMCs) as a model. The challenge with saliva collected from *Ae. albopictus* caused a significant increase of beta-hexosaminidase activity levels suggesting that cultured BMMCs degranulate in response to salivary proteins.

Based on the above finding, we next investigated the potential interactions between mast cells and two *Ae. albopictus* salivary proteins, the adenosine deaminase (ADA) and the 34k2. ADA is a metabolic enzyme with the capacity to converse the nucleosides adenosine into inosine and ammonia. ADA in insects may have an anti-inflammatory role in that adenosine can cause vasodilation and inhibit platelet aggregation [29]. The *Aedes aegypti* ADA was reported to be upregulated after blood feeding, and while it enhanced dengue virus replication it had an inhibitory effect on chikungunya virus [30–32]. The *Ae. albopictus* ADA (alADA) induced host IgG antibody production [33], and recombinant alADA has successfully been expressed [34]. 34k2, a member of the 34kDa salivary protein family, is a newly identified mosquito salivary protein. 34k2 of both *Aedes aegypti* (aa34k2) and *Ae. albopictus* (al34k2) species can induce the production of IgG antibodies [28]. Compared with aa34k2, IgG against al34k2 might be considered as a reliable candidate marker to detect the variation of human exposure to *Ae. albopictus* [27]. Tryptase and chymase were demonstrated to have the capacity to recruit leukocytes and induce vascular leakage [35–37]. In our hands, 10 μg/ml of alADA was required for significant activation of the mast cells in cell culture. Although this may be a high concentration compared with the physiological milieu at the mosquito biting site, it indicates that alADA potentially can activate mast cells *in vivo*. However, since only 10 ng/ml of saliva induced a significant mast cell activation, our result suggests that alADA together with other, as yet unknown, saliva proteins cause mast cell degranulation. We also demonstrated that both alADA and al34k2 exerted modulating roles of the enzymatic activities of the mast cell-specific proteases. However, the potential outcome *in vivo* of the described interactions between alADA and al34k2 and the mast cell-specific proteases remains to be studied.

It is well known that when activated mast cells release large amounts of mediators, including tryptase and chymase. Tryptase consists of four functional monomers stabilized by heparin, forming a tetramer with the four substrate pockets facing inwards the central ”pore”. Tryptase prefers to cut after positively charged lysine (K) or arginine (R) in its three amino acid target sites (K/R + X + K/R) [38]. Chymase is a monomeric serine proteinase and the physiologic extended target sites for chymase have been shown to be eight amino acids long (P4, P3, P2, P1, P1’, P2’, P3’, P4’). Chymase preferentially cuts after aromatic amino acids tyrosine (Y), phenylalanine (F), or tryptophan (W) located in the P1 position and often requires glutamic acid (E) or aspartic acid (D) in the P2’ position [39–41]. However, the targeted sites for degradation by chymase remain abstruse. Here we found both alADA and al34k2 contain predicted target sites for tryptase and chymase, and we showed that both rHT and rHC could degrade alADA and cleave al34k2. This suggests that the potential physiological functions of alADA and al34k2 can be timely reduced through cut by tryptase and chymase released from activated mast cells.

In summary, we here showed that *Ae. albopictus* saliva caused mast cell degranulation, a degranulation partly induced by alADA. Furthermore, we showed a direct interaction between alADA and al34k2 and the mast cell-specific proteases, as reflected by alADA- and al34k2-induced enzymatic activity modulation and the protease-dependent degradation of alADA and al34k2. Together, this suggests that alADA and al34k2 can regulate the functions of tryptase and chymase, which may have impact on the inflammatory responses induced by mosquito saliva. However, the physiological function of alADA and al34k2 can be restricted by degradation or cleavage by tryptase and chymase.

## Conclusions

This study is the first report on the functional interactions of two *Ae. albopictus* salivary gland proteins, alADA and al34k2, with mast cells and the two mast cell-specific proteases, tryptase and chymase. During interaction with these proteases, alADA and al34k2 may modulate mast cell-driven immune responses in the local skin microenvironment, affecting the recruitment of inflammatory immune cells, the induction of vascular leakage, and potentially regulating the development of inflammation at the mosquito bite site. We now aim to investigate the inflammatory roles of alADA and al34k2 *in vivo* using the chymase and tryptase-deficient mouse strains.

## Supplementary Material

Supplemental Material

## Data Availability

The data supporting the findings in our study are available from the submitting author (lzqforever@hotmail.com) and corresponding authors (zhenglingshang@gmc.edu.cn and jiahongw@gmc.edu.cn) upon reasonable request.
